The article "Visual Analysis of Nutrient Deficiency and Treatment Protocols in Bariatric Surgery Based on VOSviewer" was retracted in 2023. Reasons: unreliable results or conclusions; lack of ethics approval or compliance; concerns about the data; concerns about the peer review.

# Visual Analysis of Nutrient Deficiency and Treatment Protocols in Bariatric Surgery Based on VOSviewer

**DOI:** 10.1155/2022/8228831

**Published:** 2022-08-16

**Authors:** Jihong Tang, Mei He, Guirong Li, Juan He, Xianhua Wang, Zhuoxin Yang, HongJin Wu

**Affiliations:** ^1^School of Nursing, Chengdu Medical College, 610500, China; ^2^Nursing Department, Mianyang Central Hospital, 621000, China; ^3^President's Office, Mianyang Central Hospital, 621000, China

## Abstract

**Objective:**

To analyze the global literature on nutritional deficiencies in bariatric surgery (BS) since January 1, 1985, and to discuss the current status of research, research hotspots, and new development trend and treatment of nutritional deficiency in bariatric surgery. It provides ideas and basis for promoting the development of bariatric surgery and new alternative therapy or treatment protocols.

**Methods:**

The Web of Science (WOS) database core collection was used as the data source, and VOSviewer 1.6.17 software was used to search the literature on the topic of “nutritional deficiencies in bariatric surgery.” The number of published literature, the distribution of authors, institutions, and countries, keyword cooccurrences, and journal cocitations were visualized and analyzed.

**Results:**

A total of 1015 relevant publications was obtained after searching and screening, and the overall trend of literature published was on the rise. The most published countries, institutions, and authors were USA, University of Sao Paulo, Ramalho, Andrea; Obesity Surgery has been the most frequently cited journal (7943 citations), and the top 10 journals had high impact factors. Keyword cooccurrence analysis showed that “bariatric surgery” and “nutritional deficiencies” are the hot topics of research in this field.

**Conclusion:**

There is an urgent need for bariatric surgery issuing institutions and authors to strengthen cross-institutional, cross-team, and multicenter and multidisciplinary cooperation, to promote and facilitate the exchange and cooperation in the field of bariatric surgery between developed countries in Europe and America and developing countries in Asia, Africa, and Latin America, to draw the attention of developing countries to the health problems caused by obesity, and to encourage and support the development of developing countries in this field. Bariatric surgery, obesity, weight loss, Y-type gastric bypass, gastric bypass, and nutritional deficiency are the hot research topics in the field of nutritional deficiency in bariatric surgery, and metabolic surgery, single anastomosis gastric bypass, micronutrient supplementation, micronutrient deficiency, intestinal microbiology, and guidelines are the new trends in this field.

## 1. Introduction

Obesity is officially recognized as a global disease and a persistent risk factor for chronic diseases [1]. Obese patients are frequently accompanied by other comorbidities, such as type 2 diabetes, dyslipidemia, insulin resistance, and cardiovascular disease [2]. In 2016, more than 1.9 billion adults aged 18 years and older were overweight globally, of whom more than 650 million were obese, and 39% of adults aged 18 years and older were overweight and 13% were obese [3]. According to the World Health Organization, it is estimated that by 2025, about one-fifth of the world's adults will be obese [4]. And the Report on the Status of Nutrition and Chronic Diseases in China (2020) shows that the problem of overweight and obesity in urban and rural residents of all age groups continues to be highlighted, with more than half of the adult population being overweight and obese [5]. Options for treating obesity include three main categories: lifestyle interventions, drug therapy, and bariatric surgery. Lifestyle interventions and pharmacotherapy alone have been shown to be ineffective in sustaining weight loss [6]. The results of the study demonstrate that bariatric surgery is an effective treatment for obesity [7] and gets more attention. According to the China Bariatric Metabolic Surgery Database Annual Report 2020, the actual total number of bariatric surgery cases nationwide is projected to be about 14,037 [8], and the acceptance of bariatric surgery by the general public is gradually increasing. However, weight loss surgery has strict criteria, international recommendations for body mass index (BMI) > 40 or BMI in the range of 35-39.9 and suffer from one of the metabolic complications associated with obesity, surgery is recommended, BMI in about 30 to consider surgery [9]. According to the ethnic characteristics and differences of the East Asian population, surgery is actively recommended in China for BMI ≥ 37.5 kg/m^2^; to 32.5 kg/m^2^ ≤ BMI < 37.5 kg/m^2^, surgery is recommended; for 27.5 kg/m^2^ ≤ BMI < 32.5 kg/m^2^, which is difficult to control with lifestyle changes and medical treatment and at least 2 components of metabolic syndrome are met or comorbidities exist [10]. The two most commonly used procedures internationally are SG (sleeve gastrectomy) and Roux-en-Y-gastric bypass (RYGB) [11]; SG is done by removing approximately 80% of the size of the stomach; RYGB is a Y-shaped division of the stomach into upper and lower parts, with the small upper part anastomose with the distal small intestine and the severed proximal small intestine anastomose with the distal end laterally to form a Y shape. Both procedures achieve sustained weight loss and are also effective in the improvement of comorbidities. However, postoperative complications remain deserving of our attention. Nutritional deficiency is the most frequent postoperative complication of bariatric surgery and is associated with anemia [12], secondary hyperparathyroidism, and metabolic bone disease [13]. Nutritional deficiencies in bariatric surgery can be related to partial gastrectomy or foods, bypassing key nutrient absorption sites (e.g., duodenum/jejunum proximal), which limits dietary intake and decreases nutrient uptake [9, 14]. The results of related studies [15, 16] suggest that nutritional deficiencies in bariatric surgery can be improved through perioperative lifestyle interventions, long-term nutritional monitoring and postoperative follow-up, and increased patient awareness through a guided collaborative/participatory nurse-patient model to reduce postoperative nutritional deficiency complications and significantly improve patient compliance. VOSviewer software enables quantitative and visual analysis of knowledge structures, research hotspots, and frontiers [17]. Based on the Web of Science core collection database, this paper analyzes the current status, hotspots, and development trends of domestic and international research on nutrient deficiencies in bariatric surgery since January 1, 1985, using VOSviewer software, hoping to bring some new references and data for future research work.

## 2. Materials and Methods

### 2.1. Sources and Literature Search

The search was conducted using the core collection on the Web of Science, an English-language literature repository with a wide academic impact, as the data source, and a search strategy was constructed in the advanced search interface, including English search terms related to bariatric surgery, nutrients, and deficiencies. ((TS = (Bariatric surgery or Metabolic Surgery or Bariatric Surgical Procedures or obesity surgery or gastric bypass or sleeve gastrectomy or laparoscopic Roux-en-Y gastric bypass or laparoscopic sleeve gastrectomy or laparoscopic gastric bypass or Endoscopic weight loss surgery or adjustable gastric banding or laparoscopic adjustable gastric banding or one-anastomosis gastric bypass or mini gastric bypass or Biliopancreatic diversion with duodenal switch or duodenal-jejunal bypass or transit bipartition or jejunal-jejunal bypass or jejunoileal bypass or duodenal switch/single-anastomosis duodenoileal bypass with sleeve gastrectomy or Fundoplication or Balloon or Stomach Stapling)) AND TS = (defici∗)) AND TS = (Nutri∗))) AND DT = (Review OR Article). The search was conducted from January 1,1985, to March 13, 2022, in any language, and 1017 articles were retrieved, and 1015 valid articles were obtained by further eliminating duplicates using the EndNote Document Manager.

### 2.2. Methods and Tools

All the retrieved literature was exported; tab-delimited files were selected; information was entered as “full record with cited references” and saved as a “plain text” file in savedrecs.txt format to the specified path. By using VOSviewer 1.6.17 software, the search results were analyzed in terms of author, institution, country, keywords, and journal citations to explore the current status, trends, and hotspots in the field.

## 3. Results

### 3.1. Analysis of the Amount of Literature Published

A total of 1015 papers was collected from 1985 to March 13, 2022. As shown in Figure 1, there is an overall upward trend in the number of publications related to nutritional deficiency research on BS. From 41 articles in 2009 to 115 articles in 2021, the number of articles increased approximately 2.8 times during this twelve-year period. The number of publications showed an increasing trend from 2009 to 2020, with a small decline in 2013, 2015, and 2018, followed by a significant increase in 2020 and 2021. As of the search date of March 13, 2022, 24 articles have been published.

### 3.2. Analysis of the Distribution of Coauthors and Institutions

Visual analysis of authors and institutions was done, publication of research in the field of nutrition deficiencies in bariatric surgery. The analysis type was coauthorship, and the minimum number of publications in the default software for authors and institutions was 5. Out of 4797 authors, a total of 71 authors met this threshold, and out of 1674 institutions, a total of 97 institutions met this threshold. In the field of nutritional deficiencies in bariatric surgery, the top three authors with the most scientific publications were Ramalho, Andrea (17), Saboya, Carlos (14), and Ben-Porat, Tair (14), and the other authors with the most publications are detailed in Table 1. A total of 15 research or medical institutions had 10 or more publications, with the top three most published institutions being the University of São Paulo (29), Mayo Clinic (25), and the Assuta Medical Center (17). Refer to Table 2 for more details on the volume of articles issued by other institutions. In Figures 2 and 3, one color represents one group, and each group represents one team of authors or one institutional consortium. A collaboration between authors is primarily restricted to internal team members, and team-to-team collaboration is extremely poor, as shown in the visual analysis table of the authors' collaboration in Figure 2. There is some cooperation between the institutions, but it is still relatively limited and most of them do not cooperate with one another. The visual analysis chart of institutional cooperation is detailed in Figure 3.

### 3.3. Analysis of Country Distribution

Visualization of countries with research in the field of nutritional deficiencies in bariatric surgery was done. The analysis type is coauthorship, and the default country minimum number of publications is 5. Out of 68 countries, a total of 39 meet this threshold and the publication of scientific results is mainly concentrated in European and North American countries. The largest number was from the United States, with 348 articles or 34.28%. Although Brazil, China, and Israel also appear in the ranking, they account for a very small percentage, and the specific ranking of country issuance is detailed in Table 3. In Figure 4, there are as many as 253 connecting lines between countries, with a total linkage intensity of 546, with particularly strong links between European and American countries. The visual analysis chart of country cooperation and distribution is detailed in Figure 4.

### 3.4. Keyword Analysis

The visual analysis of keywords by VOSviewer software can reflect the hotspots and development trends in the field of malnutrition in bariatric surgery and explore potential new development directions and research hotspots in the field.  Figure 5 shows that the larger the size of the sphere, the higher the frequency of keywords and the more focused the research focus.  Figure 6 shows that the more the color of the sphere tends to be yellow, the newer the direction of research in this area is represented.  Figure 7 shows that the color brightness is positively correlated with the study hotspots. The minimum frequency of keywords was set to 5, and 351 out of 3309 keywords met the threshold requirements, and the specific results are shown in Table 4. The top 6 keywords in terms of frequency were “bariatric surgery (642)”, “obesity (371)”, “weight loss (221)”, “Y-shaped gastric fraction (221)”, and “Y-shaped gastric fraction (221)”. “Weight loss (221)”, “Y-shaped gastric bypass (220)”, “gastric bypass (193)”, and “nutrient deficiency (183)” suggest a strong relationship between nutrient deficiency and bariatric surgery, which is one of the important complications of bariatric surgery [15]. Other keywords such as “outcome”, “complications”, “anemia”, “vitamins”, and “malnutrition” indicate that postoperative complications are related to deficiencies of nutritional elements and micronutrients [12, 16]. Notably, “female” and “pregnancy” also appear in the keywords, and Mead et al. [18] showed that weight loss surgery not only affects women's nutritional deficiencies during pregnancy but also the risk of low mean birth weight of the newborn. Starting in 2019, “celiac disease”, “vitamin D supplementation”, “single anastomosis gastric bypass”, and “healthy nutrition guidelines” have become new research directions and concerns, suggesting that healthcare professionals need to pay more attention to perioperative nutritional deficiencies in bariatric surgery and take active countermeasures to correct and improve them. A visualization of the coverage of keywords evolving over time is shown in Figure 6.

### 3.5. Journal Cocitation Analysis

A cocitation analysis of the source journals for literature related to nutritional deficiencies in bariatric surgery showed that the top three journals cited were Obesity Surgery, Surgery for Obesity and Related Diseases, and American Journal of Clinical Nutrition. The quality of the journals is relatively high in terms of citation counts and impact factors, and research on nutritional deficiencies in bariatric surgery has entered a phase of high-quality research and is receiving increasing attention. The journal citation rankings are detailed in Table 5. The connectivity between different journals is dense, and the journals are more closely linked to each other. Visual analysis of journal cocitations is shown in Figure 8.

## 4. Conclusion

An analysis of the literature on nutritional deficiencies in bariatric surgery included in the Web of Science database since January 1, 1985, showed an overall upward trend in the number of articles published. During this period, research on nutritional deficiencies in bariatric surgery developed rapidly and achieved remarkable results. Ramalho, Andrea was the most published author whose research focuses on the complications associated with micronutrient deficiencies in women, pregnancy, and bariatric surgery. While the United States, France, Brazil, the United Kingdom, and Italy are the five countries with the highest number of publications, the University of São Paulo, Mayo Clinic, and Assuta Medical Center are the main research institutions that are leaders in the field with their comprehensive and in-depth research in the area of nutritional deficiencies in bariatric surgery.

Analysis of the degree of cooperation between author groups and publishing institutions provides an overall picture of the depth and breadth of research activities in related fields [19]. The analysis of the distribution of authors, institutions, and countries shows that the authors of studies on nutritional deficiencies in bariatric surgery come from different countries, indicating that the problem of nutritional deficiencies in bariatric surgery has gradually started to receive continuous attention in various countries around the world and is being studied in depth with “globalization” and scientific and technological advances. There is also a degree of exchange and cooperation between research or medical institutions in different countries and regions. This indicates that the problem of nutritional deficiencies in obesity and bariatric surgery is no longer a regional or local problem, but a global one that is difficult to solve on its own and requires the search for cooperation and win-win solutions. The visual analysis of authors and institutions in maps shows that the authors have many teams that work closely together and have developed a large influence, but the collaboration between authors is mostly limited to within teams, and there is almost no collaboration between teams. At the same time, cooperation among agencies is fragmented and less continuous, with a few agencies working closely with each other, but mostly as different units under the same agency. It may be related to geographic restrictions, especially after COVID-19, when countries have intensified the difficulty of cross-regional and cross-country communication and cooperation due to epidemic prevention and control requirements. From the visual analysis of the country distribution, it is known that the research results on nutritional deficiencies in bariatric surgery are mainly concentrated in Europe and North America, with a significantly higher number of Western European countries than Southern Europe, which may be related to the culture and eating habits of the Southern European diet (Mediterranean diet [20]). There are very few developing countries conducting research and producing scientific results in the field of weight loss, mainly in Asia and South America, probably influenced by the level of economic development and traditional culture, with less research on metabolic surgery nutritional deficiencies and less exchange and cooperation in this field with developed countries in Europe and America. However, it is interesting to note that Brazil and China are the 3rd and 13th countries, respectively, in terms of scientific publications in the field of nutritional deficiencies in bariatric surgery. This may be related to two things. (1) With the rapid economic development, the fast pace of life and work, and the advancement of mobile payment technology, the takeout industry relying on major technology platforms is gradually becoming popular and blooming among young people, especially in the postepidemic era [21]. While technology has brought about the ability to enjoy food without leaving home, dietary patterns and habits are quietly changing, with a preference for diets or beverages high in fat, oil, salt, and sugar and a decreasing willingness to exercise, leading to a rapid increase in the number of obese people [22]. In addition, young people work and study under pressure [23] and often stay up late [24, 25]; these unhealthy lifestyles also caused the growth of the number of obesity. (2) In the field of bariatric surgery, although Brazil and China started late, they had a high starting point. With the popularization of laparoscopic technology and minimally invasive surgery concept, BS is gradually becoming familiar to the public, and more and more people are undergoing BS. Therefore, when facing the health problems caused by obesity and the problem of nutritional deficiency after bariatric surgery, the whole world should unite to actively deal with it, start an ice-breaking action, remove barriers, adopt the methods of online network meetings and offline experience exchange and sharing, and strengthen the communication and cooperation among transnational, cross-regional, cross-center, and cross-institution, to allow more obese patients to gain health.

Analysis of the keyword network shared knowledge graph revealed that the hotspots of research on nutritional deficiencies in bariatric surgery can be broadly classified into 4 categories: (1) keywords that reflect the type of obesity are obese and morbid-obesity; (2) the keywords that reflect the type of treatment are bariatric surgery, weight loss, Y gastric bypass, gastric bypass, sleeve gastrectomy, biliopancreatic diversion, surgery, gastric-bypass surgery, Roux-en-Y gastric bypass, and laparoscopic sleeve gastrectomy; (3) the keywords that reflect the type of postoperative outcome are nutritional deficiencies, outcomes, deficiency, complications, deficiencies, anemia, and malnutrition; (4) keywords that reflect the type of postoperative nutritional management. Among them, “bariatric surgery”, “obesity”, “weight loss”, “Y-shaped gastric bypass”, “gastric bypass”, and “nutritional deficiency” are the keywords that appear most frequently and become the hotspots of research, indicating that surgical treatment of obesity is gradually becoming mainstream. Still, the problem of postoperative nutritional deficiency is also becoming more and more prominent, which requires bariatric surgeons and researchers to jointly explore the mechanisms and causes behind its occurrence and find treatment methods from the root. Other keywords such as “outcome”, “complications”, “anemia”, “vitamins”, and “malnutrition” suggest a link between nutritional deficiency as an adverse outcome after bariatric surgery and other related complications. It is recommended [26] that a multidisciplinary collaborative and integrated treatment and treatment model of perioperative nutritional management throughout the process of preoperative assessment, intraoperative monitoring, postoperative rehabilitation, and postoperative follow-up can effectively alleviate and prevent perioperative nutrient deficiencies in bariatric surgery.

In addition, Smelt et al. [27] showed that specific bariatric multivitamins targeted for individualization can improve micronutrient deficiencies. It is noteworthy that more and more authors are becoming concerned about the impact of BS of nutrient deficiencies in women during pregnancy, early/recurrent miscarriage, and low birth weight in newborns [18, 26]. Guidelines recommend that the provision of nutritional supplementation and close monitoring can be effective in improving nutritional deficiencies and generating good pregnancy outcomes [18, 28]. Starting in 2019, new keywords such as “celiac disease” [29], “vitamin D supplementation” [30–32], “single anastomosis gastric bypass” [33–36], and “healthy nutrition guidelines” [15] are gradually appearing more frequently in studies on nutritional deficiencies in BS. This indicates that researchers are not only concerned about macronutrient deficiencies but also about micronutrient deficiencies; at the same time, they are actively exploring surgical procedures that are simpler and less invasive and avoid postoperative complications such as nutritional deficiencies.

From the analysis of journal cocitations, currently, the research results published in the field of bariatric surgery are mainly in international journals such as Obesity Surgery, Surgery for Obesity and Related Diseases, and American Journal of Clinical Nutrition, which also includes top international journals such as New England Journal of Medicine and JAMA—Journal of the American Medical Association. From a side viewpoint, the problem of bariatric surgery and postoperative nutritional deficiencies has been paid attention by more and more authors and has been thoroughly analyzed and studied [37]. Bariatric surgery has been shown to be a safe, cost-effective, and sustainable approach to weight loss [38, 39], but only a small percentage of the population can actually benefit from it [40]. In addition, the acceptance of and access to bariatric surgery varies from country to country depending on the country's level of economic development and traditional beliefs. As the world's most populous country, China has the highest total number of obese people in the world [5]. There were 9839 bariatric procedures in China in 2018, accounting for only 1.4% of the total worldwide (696,191) [11]. According to statistics, there will be about 14,037 bariatric surgeries in China in 2020 [8], an increase of 42.7% compared to 2018, but the percentage is still very low compared to the total obese population in China. This may be related to the traditional perception that Chinese people prefer to receive medical treatment. As the world's largest developing country, China has a relatively high level of national economy, but with a large population and low per capita income level, coupled with the fact that obesity is not currently considered a disease in China and is not covered by medical insurance, the vast majority of patients who want to reduce their weight through surgery are turned away. The late start of bariatric surgery in China, the lack of data, and the relative lag in research have resulted in significantly fewer research results being published in international high-quality journals than in developed countries in Europe and the United States. As a non-English speaking country, most authors also prefer to publish their research in Chinese domestic journals, which to some extent diminishes the international influence of China in the field of bariatric surgery. In order to eliminate the large number of obese people in China as soon as possible, it is recommended that China adopt a strategic approach of “bringing in” and “going out.” “Bringing in” is based on China's established bariatric surgery database, introducing advanced international technology and equipment and concepts, employing full-time bariatric surgeons and bariatric case managers, and combining MDT teams to improve surgical quality and safety while reducing postoperative complications. “Going out” is to strengthen exchanges and cooperation with developing countries in the field of bariatric surgery, such as visiting schools, attending conferences, and exchanging experiences, so as to produce more high-quality clinical research results and improve medical quality and clinical efficacy for the benefit of patients.

## 5. Summary

This study visualized and analyzed the collected literature on nutritional deficiencies in bariatric surgery from multiple perspectives by using VOSviewer software to derive the current status of research, research hotspots, and new research trends in this field and to actively explore possible new treatment options for future new treatment protocols. Nutritional deficiencies in bariatric surgery have received widespread attention from scholars around the world, with closer collaboration between institutions than between authors, but there is an urgent need for cross-institutional, cross-team, and cross-national academic exchange and collaboration between authors, institutions, and countries. The WOS Core Collection database is an authoritative database of academic information worldwide, which includes important academic journals and international conferences worldwide with a strict screening mechanism, and the literature included in WOS belongs to the type supported by the operation of VOSviewer software, so the literature from the WOS Core Collection database was selected for analysis. Multidatabase analysis was not conducted in this study, which has the defect of incomplete data, and multidatabase analysis will be conducted in other studies in the future.

## Figures and Tables

**Figure 1:** Literature publications.

**Figure 2:** Analysis of coauthor distribution.

**Figure 3:** Analysis of the institutional distribution of coauthors.

**Figure 4:** Analysis of the country distribution of coauthors.

**Figure 5:** Frequency analysis of keyword occurrence.

**Figure 6:** Analysis of changes in keywords by year.

**Figure 7:** Analysis of keyword hotspot.

**Figure 8:** Analysis of journal cocitation.

**Table 1:** Ranking of authors with 10 or more publications.

Institution	Documents	Citations	Total link strength
Ramalho, Andrea	17	185	40
Saboya, Carlos	14	151	39
Ben-Porat, Tair	14	260	37
Pereira, Silvia	11	119	35
Aarts, Edo, O.	11	340	21
Sherf-dagan, Shiri	10	34	34
Coupaye, Muriel	10	385	25
Kaifarentzos, Fotis	10	489	4

**Table 2:** Ranking of institutions with 10 or more publications.

Institution	Documents	Citations	Total link strength
Univ Sao Paulo	29	612	5
Mayo Clin	25	2404	27
Assuta Med Ctr	17	242	64
Katholieke Univ Leuven	15	1038	13
Univ Fed Rio de Janeiro	15	187	3
Hebrew Univ Jerusalem	13	273	41
Univ Minnesota	13	824	12
Rijnstate Hosp	13	444	9
Hadassah Hebrew Univ	12	269	34
Brigham & Women's Hosp	12	613	9
Harvard Med Sch	11	151	11
Harvard Univ	10	1306	33
Hadassah Hebrew Univ Med Ctr	10	124	22
Univ Hosp Leuven	10	297	8
Med Univ Vienna	10	1924	6

**Table 3:** Top 15 ranking of coauthors' countries in terms of number of publications.

Country	Number of articles published	Percentage
USA	348	34.28%
France	91	8.97%
Brazil	83	8.2%
UK	68	6.7%
Italy	64	6.3%
Spain	60	5.9%
Germany	49	4.8%
Netherlands	43	4.2%
Canada	41	4.0%
Australia	39	3.8%
Belgium	35	3.4%
Israel	35	3.4%
China	30	3.0%%
Switzerland	28	2.8%
Greek	25	2.4%

**Table 4:** Frequency of keywords.

Keywords	Frequency of occurrence	Total linkage strength
Bariatric surgery	642	5149
Obesity	371	3071
Weight loss	221	1949
Y gastric bypass	220	1964
Gastric bypass	193	1601
Nutritional deficiencies	183	1590
Sleeve gastrectomy	160	1440
Morbid-obesity	130	1203
Biliopancreatic diversion	117	1081
Outcomes	106	882
Deficiency	100	767
Complications	93	781
Surgery	85	626
Nutrition	79	643
Gastric-bypass surgery	78	672
Deficiencies	78	632
Guidelines	76	698
Roux-en-Y gastric bypass	76	685
Anemia	73	679
Follow-up	71	663
Malnutrition	70	592
Laparoscopic sleeve gastrectomy	66	636
Women	66	591
Prevalence	66	573
Pregnancy	65	582
Vitamin	64	600

**Table 5:** Journal citations and impact factor.

Citation ranking	Journal name	Citations	Impact factor
1	Obesity Surgery	7943	4.1291
2	Surgery for Obesity and Related Diseases	2901	4.734
3	American Journal of Clinical Nutrition	1357	7.047
4	New England Journal of Medicine	1074	91.253
5	Annals of Surgery	948	12.970
6	JAMA—Journal of the American Medical Association	836	56.274
7	Journal of Clinical Endocrinology & Metabolism	831	5.958
8	Obesity	645	5.002
9	International Journal of Obesity	550	5.095
10	Clinical Nutrition	541	7.325

## Data Availability

The data used to support the findings of this study are included within the article.
